This article has been retracted.

# Molecular insights into the anti-cancer properties of Traditional Tibetan medicine *Yukyung Karne*

**DOI:** 10.1186/1472-6882-14-380

**Published:** 2014-10-07

**Authors:** Tenzin Choedon, Dawa Dolma, Ganeshan Mathan, Vijay Kumar

**Affiliations:** Virology Group, International Centre for Genetic Engineering and Biotechnology, Aruna Asaf Ali Marg, New Delhi, 110067 India; Department of Biomedical Science, Bharathidasan University, Tiruchirappalli, 620024 India; Tibetan Medical Astro Institute, Dharamsala, Kangra 176215 India

**Keywords:** *Yukyung Karne*, Traditional Tibetan medicine, Ovarian cancer, Apoptosis, Mitochondria membrane potential

## Abstract

**Background:**

*Yukyung karne (YK)* is a traditional Tibetan formulation used for many centuries for the treatment of ovarian cancer. However, the pharmacological basis of its anticancer property is not well understood. In the present study, the anticancer property of YK was investigated in cell culture.

**Methods:**

The growth inhibitory property of *YK* was evaluated in SKOV6, IHH, HepG2 and HEK293 cell lines using MTT assay. The pro-apoptotic activity of drug was analyzed by terminal deoxynuleotidyl transferase dUTP nick end labeling (TUNEL) and DNA fragmentation assays. Confocal microscopy was used to show the release of cytochrome c and its co-localization with mitochondria with the help of dsRed mitotracker in SKOV6 cells. The inhibition in cell proliferation was also visualized by confocal microscopy after BrDU incorporation. The activation of tumor suppressor p53 was evaluated by Western blotting while VEGF levels in culture supernatant were measured by a colorimetric method.

**Results:**

*YK* specifically and efficiently induced apoptotic killing of the human ovarian cancer SKOV6 cells as indicated by increased DNA fragmentation and nick end DNA labeling. Confocal microscopy suggested inhibition of cell proliferation and increase in cytochrome c release via perturbation in mitochondrial membrane potential (Δψm). Further, *YK* up-regulated the expression of tumor suppressor p53 and key cyclin-dependent kinase inhibitor p21, and inhibited VEGF secretion by cells. Interestingly, *YK* also exhibited a synergy with paclitaxel which is a well-known anti-cancer therapeutic drug.

**Conclusions:**

The pharmacological properties of *YK* to impose growth arrest and trigger pro-apoptotic death in cells amply justify its usage in primary as well as adjunct therapy for ovarian cancer.

**Electronic supplementary material:**

The online version of this article (doi:10.1186/1472-6882-14-380) contains supplementary material, which is available to authorized users.

## Background

Ovarian cancer is one of the most lethal gynecological malignancies and a leading cause of cancer related death in women [1]. The conventional treatment regimen for ovarian cancer includes combination of platinum based chemotherapy, surgery and radiation [2]. However, none of these therapies have impacted the overall survival rate significantly [3]. Despite several advancements made during past few decades, there is enough scope for developing new methods and therapeutic agents for effective treatment of ovarian cancer.

Natural products are excellent sources of complex chemicals with useful properties including great therapeutic value [4]. Dietary phytochemicals such as curcumin [5] and Silibinin [6] have been identified as two major natural anticancer agents. Curcumin and Silibinin have been extensively used in the traditional medical system in Asia. Traditional Tibetan medicine (TTM) with over 2000 years old legacy of holistic and naturopathic approach integrates diet, behaviour, lifestyle, herbs and accessory therapies are integrated to treat the root cause of disease [7]. The main constituents of the Tibetan medicine are *Terminalia chebula (Aru ra), Terminalia belerica (Baru ra)* and *Emblica officanalis* (*Kyuru ra*) popularly known in Tibetan as *Aru-Baru-Kyuru* in a ratio of 2:1:1 just as Triphala in Ayurveda [8]. TTM are mostly multi-ingredient formulation comprising 3 to 150 herbs and minerals to combat multifactorial diseases like cancer [9]. Many Tibetan medicines are considered safe, effective, non-toxic and most of all good therapeutic value for a number of chronic diseases [10–12]. Earlier we reported that Thapring, a TTM used for the treatment of chronic liver diseases, can inhibit cell proliferation and induce apoptosis in a transgenic mouse model of hepatocellular carcinoma [13]. Since ovarian cancer is difficult to treat and relapse rate is quite high, many patients opt for complementary therapy to ease stress, symptoms and better survival. Interestingly, the therapeutic response of another TTM formulation -*Yukyung Karne* (*YK*) [14] has shown promising results by providing relief to the ovarian cancer patients. In the present study, we provide evidence based mechanistic insights into the anticancer properties of *YK*.

## Methods

### Chemicals, reagents and kits

Paclitaxel was purchased from Calbiochem, Propidium iodide, methanol, DMSO and 3-[4,5-dimethylthiazol-2-yl]-2,5 diphenyltetrazolium bromide (MTT) reagents were procured from Sigma Aldrich. DeadEnd Fluorometric TUNEL system was from Promega. JC1dye-5,5′,6,′-tetrachloro-1, 1′, 3, 3′ tetraethylbenzimidazolylcarbocyanine iodide was from Molecular Probes Inc., Eugene, USA. Enhanced chemiluminescence (ECL) reagent and antibodies were from Santa Cruz, USA while the VEGF quantikine ELISA kit was from R& D system (Minneapolis, USA). Dulbecco-modified Eagle’s medium (DMEM), fetal bovine serum (FBS), streptomycin and penicillin were from Gibco-BRL, USA. Lipofectamine 2000 was from Invitrogen, USA while the BrdU labeling kit was from Roche Diagnostics, Indianapolis, USA.

### Plant material

*Yukyung karne* was purchased from the Tibetan Medical and Astrological Institute (TMAI), Dharamshala, India. *YK* was dissolved in glass-distilled water and diluted appropriately for use in our experiments. No extraction step was involved. According to Tibetan Pharmacopeia [14], *YK* comprises of a mixture of root of *Saussurea lappa* (C.B. Clarke) (family: Asteraceae), fruit of *Emblica Officinalis* (L) (family: Euphorbiaceae), leaves of *Adhatoda vasica* (NEES) (family: Acanthaceae), seeds of *Elletra cardomomum* (L) (family: Zingiberaceae), fruit of *Piper longum* (L) (family: Piperaceae), whole plant part of *Dracocephyllum tanguticum* (Maxim) (family: Lamiaceae), root of *Zingiber officinalis* (Roscoe) (family: Zingiberaceae), seed of *Coriandrum sativum* (L) (family: Apiaceae), whole plant of *Meconopsis horridula (Hook)* (Papaveraceae), root of *Corydalis hendersoni* (Fedde) (family: Fumariaceae), seeds of *Embelia ribes* (Burm. F) (Family:Myrsinaceae), *Delphinium brunonianum* (Royale) (family: Ranunculaceae), fruit of *Terminalia chebula* (Rety) (family: Combretaceae), root of *Acorus calamus (*L) (family: Araceae), root of *Aconitum ferox* (Wall.ex Ser) (family: Ranunculaceae), resin of *Commiphora mukul* (Hook) (family: Burseraceae) and a mineral ingredient. All the herbs were identified by Dr. Tsering Norbu (Menrampa) and the voucher numbers of plant specimens are available at the herbarium department of TMAI for reference.

### Cell culture and transfection

Ovarian cancer cell line SKOV6 was a kind gift of Dr. Anil Suri (National Institute of Immunology, New Delhi). The human hepatoma cells Huh7 was a kind gift from Dr. A. Siddiqui (University of Colorado, Denver). The immortalized human hepatocytes (IHH) were kindly provided by Dr. F. Danniel, Institut National de la Santé et de la Recherche Médicale Unite 481, Universite Paris 7, Paris, France. HepG2, HEK 293 (CRL-1573) and A549 (CCL-185) cells were purchased from ATCC. All cultures were grown in DMEM supplemented with 10% FBS, penicillin 100 μg/ml and streptomycin (100 μg/ml) incubated at 37°C in a humidified chamber and 5% CO_2_ atmosphere. Cells were seeded at a density of 0.6 million per 60 mm dish and transfected using Lipofectamine 2000 (Invitrogen) as per manufacturer’s protocol. For tracking cytochrome c localization, pEGFP-cytochrome c (1 μg) was co-transfected with pDsRed Mitotracker (1 μg) and analyzed by confocal microscopy (Nikon A1R) Japan.

### MTT assay

Cell viability was analyzed by MTT colorimetric assay as described by van de Loosdrecht et al. [15]. Briefly, cells were seeded at density of 0.4 × 10^6^ cells per 60 mm dish, allowed to settle overnight and treated with different concentrations of *YK* (1, 10, 100 μg/ml) for 24 h. Cells were washed with DMEM without phenol red and incubated with MTT reagent for 45 min at 37°C in dark. The formazon crystals were solubilized in dimethyl sulfoxide and the absorbance was recorded at 560 nm. Untreated cells were used as control of viability (100%). The mean absorbance values of three experiments were expressed as percentage of viability in relative to control.

### Cell proliferation assay

The BrdU incorporation assay was performed using BrdU labelling kit (Roche Diagnostics, Indianapolis, IN, USA) as per manufacturer’s protocol. Nuclei were stained with DAPI (blue) while the BrdU incorporation was detected using goat anti-mouse-conjugated to FITC (green). The distribution of BrdU positive cells was shown as bar diagrams.

### Detection of DNA fragmentation

Cells were treated with different concentrations of *YK* for 24 h. Assay was carried out as per Peng et al. [16]. Briefly cells were harvested and treated with 100 μl lysis buffer and the supernatant was incubated for 2 h with RNase A at 56°C and followed by Proteinase K digestion at 37°C for 2 h. DNA was precipitated with 2.5 volume of cold absolute ethanol. The DNA pellet was dissolved in TE buffer and resolved by electrophoresis in a 2% agarose gel.

### Cell cycle analysis by FACS

Equal number of cells (0.6-0.8 × 10^6^) were seeded in each 60 mm dish and after 24 h were treated with *YK* (100 μg/ml). Cell cycle analysis was performed as mentioned by Mukherji et al. [17]. Briefly cells were fixed and stained with propidium iodide solution (50 μg/ml PI, 10 μg/ml RNase) and the data was acquired using a FACScan flow cytometer equipped with CellQuest software (Becton Dickinson, San Jose, CA, USA).

### TUNEL assay

SKOV6 cells were treated with *YK* and the level of apoptosis was detected by TUNEL assay using DeadEnd^TM^ Flourometric TUNEL kit (Promega). The assay was done as per manufacturer’s protocol. Cells were mounted using Antifade with DAPI and detected localized green fluorescence of apoptotic cells by confocal microscopy (Nikon A1R) Japan.

### Determination of mitochondrial membrane potential (ΔΨm)

For analysis of mitochondrial membrane potential, cells were seeded in 12 well plate overnight followed by treatment with *YK* for another 24 h and then stained with JC1 dye for 15 min at 37°C in 5% CO_2_ incubator. Cells were mounted with antifade mounting medium (Invitrogen, USA) and visualized at 488 nm and 590 nm using confocal microscopy (Nikon A1R) Japan.

### Estimation of vascular endothelial growth factor (VEGF)

The VEGF levels were measured as per manufacturer’s protocol (R&D system, Minneapolis). Briefly, supernatant of the experimental set of cultured cells were collected for VEGF assay. Each well was washed with wash buffer and 100 μl of the VEGF conjugate was added to each well. After repeated washing step, 100 μl of substrate solution was added to each well followed by addition of 100 μl of stop solution and mixed it gently. The OD was measured at 450 nm.

### High performance liquid chromatography (HPLC)

The fingerprints of *YK* samples were monitored on a Shimadzu reverse-phase HPLC system (C18 column - 250 mm, 4.6 mm) with SCl-10AVp system controller and SPD-10AVvp UV–vis detector. The mobile phase (acetonitrile and water) was degassed and filtered through 0.2 μm membrane filter before pumping into the HPLC system. A linear gradient of acetonitrile from 5% to 95% over 55 min at a flow rate of 1 ml/min was maintained and the samples were monitored at 220 and 280 nm using Photo Diode Array (PDA) detector. The *YK* samples (20 μg in 200 μl of glass distilled water) were used for injection.

### Western blotting

Cell lysates were prepared in cell lysis buffer. (Promega, USA) Protein concentration was determined by Bradford method. Samples with equal amounts of protein were prepared in 2x sample loading buffer (100 mM Tris–HCl pH6.8, 200 mM dithiothreitol, 4% SDS, 0.2% bromophenol blue and 20% glycerol) and resolved on 10-15% SDS-PAGE. The protein bands were visualized using the Enhanced chemiluminescent reagent (Santa Cruz, USA) according to supplier’s protocol and the image captured by Fluorchem M (Protein Simple, USA).

### Statistical analysis

Statistical significance of results in Tables 1 and 2 were calculated by Duncan’s test using SPSS software (Version 17). All other data were analyzed by Student’s *t* test. p value <0.05 was considered as significant.

**Table 1:** **Effect of** ***YK*** **on VEGF secretion from SKOV6 cells**

Sample	VEGF ± SEM (pg/ml)
Control	2.6 ± 0.057
Paclitaxel	2.10 ± 0.01*
Paclitaxel + YK	1.84 ± 0.02*
YK	1.53 ± 0.05*

*, Level of significance p Value <0.001.

**Table 2:** **Effect of anticancer drugs on cell cycle progression of SKOV6 cells**

***Sample***	***G1***	***S***	***G2***
Control	59.63 ± 2.0	17.58 ± 2.8	17.83 ± 1.09
Paclitaxel	35.0 ± 9.07*	16.65 ± 2.34	19.93 ± 3.3
Paclitaxel + *YK*	38.6 ± 6.38*	17.0 ± 1.5	18.18 ± 3.8
*YK*	73.4 ± 1.5	15.46 ± 3.09	14.18 ± 0.64

*, Level of significance: p Value < 0.004 v. control.

## Results

### Induction of apoptosis in ovarian cancer cells

An important challenge faced in chemotherapy is the adverse effect of drugs on the normal healthy cells. Most of the anticancer treatment regimen affects both cancerous as well as healthy cells. In order to establish the specificity of *YK* for ovarian cancer, we examined its effect on various cell lines by MTT assay. As shown in Figure 1A, we observed a selective induction of cell death by *YK* in ovarian and cervical cancer cell lines (SKOV6 and HeLa cells respectively). Interestingly *YK* did not induce apoptosis in IHH cells indicative of its specificity to target cancerous cells. Since *YK* exhibited a dramatic cytotoxic effect on SKOV6 cell line, it was selected for further studies. Paclitaxel a commonly used anticancer drug was used as a reference drug. As shown in Figure 1B, cells treated with paclitaxel (10 nM) showed a significant increase in cell death (p <0.005). Further MTT assay showed that treatment of *YK* in combination with paclitaxel augmented the apoptotic response induced by paclitaxel alone (Figure 1B). Since DNA fragmentation is a hallmark characteristic feature of apoptosis, we performed DNA fragmentation assay on the *YK* treated SKOV6 cells. As a noticeable fragmentation of DNA was seen at 100 μg/ml of *YK* (Figure 2A), all subsequent experiments were carried out at this concentration. We also performed TUNEL assay to confirm the observation on *YK* induced apoptosis of SKOV6 cells. As shown in Figure 2B, a significant number of TUNEL positive cells were detected in the *YK* treated cells (p <0.001) whereas no TUNEL positive cells were observed in untreated control SKOV6 cells. These data confirmed the apoptotic action of *YK* on ovarian cancer cell line.

**Figure 1:** **Growth inhibitory effect of YK on different cell lines. A**. HEK293T, A549, HepG2, Hela, IHH and SKOV6 cells were treated with different doses of *YK* (1, 10, 100 μg/ml) and analyzed for cell viability by MTT assay. **B**. SKOV6 cells was treated with *YK* and/ or paclitaxel (10 nM) and the cell viability was measured as above. Results are represented as mean of three independent experiments ± S.E.M. Level of significance; *, p <0.005.

**Figure 2:** **Induction of apoptosis by** ***YK*** **in SKOV6 ovarian cells. A**, Cells were treated with indicated doses of YK and/or paclitaxel [Lanes: 1-Control, 2-Paclitaxel 10nM, 3-Pac + *YK* (10nM + 100 μg/ml), 4–7 YK (1, 10, 100, and 200 μg/ml respectively) and 8-50 bp ladder] for 24 h. Genomic DNA was isolated and resolved by agarose gel electrophoresis. **B**, Cells were treated with different doses of *YK* (1, 10, 100 μg/ml) was visualized by TUNEL assay. The TUNEL positive cells (stained by FITC) were counted from random fields and are presented in the graph. Nuclei were visualized by DAPI staining (blue). Results are represented as mean of three independent experiments ± SD. Level of significance; *, p <0.001. **C**, Induction of cell cycle regulators. SKOV6 cells were treated for 24 h with YK (100 μg/ml), Paclitaxel (Pac) (10 μM) or both and the expression of p21, p53, Mdm2, cyclin B1, and PCNA was verified by western blot. GAPDH was used as internal control.

### Induction of tumor suppressors and cell cycle regulators

Given the key role of p53 as tumor suppressor protein in cancer prevention [18], we also studied the ability of *YK* to enhance p53 expression in the treated cells. Paclitaxel, a well-known therapeutic anticancer drug, was included as positive control as well as to evaluate its synergy with *YK*. We observed a marked increase in the cellular p53 levels after *YK* treatment (Figure 2C). However, the level of Mdm2 was down-regulated leading to the stabilization of p53. Just as p53, we also observed up regulation of pTEN, a potent tumor suppressor and p21, a potent inhibitor of cell proliferation and replication (Figure 2C). These results were further complemented by decrease in proliferation marker PCNA and cell cycle regulator cyclin B suggesting reduced proliferation of SKOV6 cells upon *YK* treatment (Figure 2C). Thus, p53 the most appealing target for mechanism-driven anticancer drug discovery, also appeared to play an important role in *YK* induced killing of cancer cell. Further, restoration of p53 functions in cancer cells by *YK* treatment could be an important strategy to combat cancer.

### Role of mitochondria-dependent intrinsic pathway in apoptosis

Since, mitochondria plays a key role in energy metabolism, and proving to be the novel target in killing cancerous cells [19], we sought to determine the effect of *YK* on mitochondrial function with the help of cationic JC1 dye. Exposure of cells to *YK* led to the disappearance of red fluorescence and increase in the green fluorescence in most cells combined with a significant reduction (p <0.001) in mitochondrial membrane potential. (Figure 3A) Further, *YK* along with Paclitaxel perturbed mitochondrial membrane potential to a significant level (p <0.05) as compared to only paclitaxel treatment (Figure 3B).

**Figure 3:** **Alterations in mitochondrial functions following** ***YK*** **treatment of SKOV6 cells. A**, Confocal images of JC1 stained cells treated with *YK* for 24 h. The green fluorescence shows depolarized mitochondria (monomer), whereas red fluorescence shows hyperpolarized (aggregates) mitochondria. **B**, Cells treated with *YK* for 24 h showing the release of cytochrome c from mitochondria during apoptosis. Cells were co-transfected with cytochrome c-GFP fusion construct and dsRed mitotracker and visualized by confocal microscopy. Green represents cytochrome c, red mitochondria and orange indicates co-localization of cytochrome c and mitochondria. Results in both panels are represented as mean of three independent experiments ± SD Level of significance; *, p <0.05; **, p <0.001.

Since release of cytochrome c from depolarized mitochondria and binding to Apaf1 are crucial steps in the formation of apoptosome, next we monitored the release of GFP-tagged cytochrome c from *YK* treated SKOV6 cells by confocal microscopy. Interestingly a significant increase was observed in cytochrome c released from dsRed Mitotracker-tagged mitochondria as indicated by a significant decrease (p <0.001) in co-localization of cytochrome c (GFP) with Mitochondria (dsRed) (Figure 3B). Taken together, these observations suggested that the mitochondria-dependent intrinsic apoptotic pathway is involved in *YK-*induced cell death.

### Anti angiogenic effect of YK

Sustained angiogenesis is another hallmark of cancer. Neo-angiogenesis is essential for supplying nutrients to the fast growing cancerous cells. Therefore starving the cancer cells is one of the most promising approach to fight cancer [20]. Of various growth factors that regulate angiogenesis, VEGF is believed to be the most important factor. To explore if *YK* could block angiogenesis, we used ELISA to measure the levels of VEGF secreted by the *YK* treated cells. Duncan analysis of these results (Table 1) revealed that all the four groups were significantly different from each other and that the VEGF levels in treated groups were lower than control (p <0.05).

Another most prominent change seen in cancer is the deregulation of cell cycle [21]. Anticancer agents on the other hand, may exert their effect by halting the cell cycle progression [22]. Therefore, next we studied the cell cycle distribution of SKOV6 cells treated with *YK* by FACS. Duncan test revealed that two groups of significant difference exist. The paclitaxel- and paclitaxel + YK-treated groups are not different from each other but are different from control- and *YK*-treated groups in the cells of G1 phase (p <0.05). Further, the control and *YK* groups are not different from each other. No significant difference was observed in four groups of cells of S and G2 phases.

Since, *YK* could abrogate cell cycle progression we also checked cell proliferation status using BrdU incorporation. *YK* treatment led to a significant reduction in the number of the BrdU positive cells. Further combined treatment with *YK* and paclitaxel showed the maximum reduction in proliferating cells. (Figure 4B) Together, these observations suggested that *YK* can inhibit proliferation by inducing cell cycle arrest at G1 phase and thus could be useful as an effective anticancer agent.

**Figure 4:** **Inhibition of cell proliferation in the presence of** ***YK.*** SKOV 6 cells were treated with paclitaxel (10nM) and/or *YK* 100 μg/ml for 24 h and analyzed by confocal microscopy for BrdU incorporation for DNA synthesis. Results are represented as mean of three independent experiments ± SD. Level of significance; *, p <0.02, **, p <0.002.

## Discussion

Despite significant advances made in the area of cancer chemotherapy, chemo resistance continues to be a major problem associated with the outcome of treatment [23]. Further, efficient targeting of cancer cells still remains a major challenge for the scientists. Therapies which are capable of inducing selective apoptosis in cancer cells are gaining attention as new potential alternative. The conventional treatment for ovarian cancer includes the administration of paclitaxel or cisplatin as a standard postoperative chemotherapy for advanced cancer patients [24], but the adverse effects are often inevitable. In this report, we provide a scientific basis for the clinical outcome of *YK*, a TTM that has been used in regular clinical practice for targeted therapy of ovarian cancer. Besides we studied the complementary action of *YK* with a well-known anticancer drug paclitaxel. We found that *YK* can induce cytotoxicity specifically in cancer cells and spared immortalized cell lines such as IHH. The *YK-* treated cells exhibited typical characteristic of apoptosis such as DNA fragmentation and apoptotic cell death as evident from the MTT and TUNEL assays (Figures 1 and 2).

Given the central role of mitochondria in initiating the apoptotic process by releasing cytochrome c, we studied the effect of *YK* on mitochondria and asked if the *YK*-induced apoptosis was mitochondria dependent. We observed that *YK* perturbed the mitochondrial membrane potential which triggered the release of cytochrome c which in turn activated the apoptotic machinery [25].

One of the key mechanisms of action of anticancer drug on cell is to halt cell cycle progression [26]. We also investigated the effect of *YK* on cell cycle progression in cancer cells by FACS analysis. Interestingly, we found that treatment with *YK* led to the arrest of SKOV 6 cells in G1 phase suggesting its growth inhibitory property (Figure 4A). This was further supported by the down regulation of cyclin B in the *YK-* treated cells which otherwise allows the cell cycle progression to S phase. Nevertheless, these results did not rule out the possibility of activation of some crucial cell cycle checkpoint inhibitors in the treated cells in order to prevent their proliferation. In this context it was interesting to observe the restoration of p53 levels in the *YK*-treated cells which may be responsible for their G1 arrest as also supported by the down regulation of PCNA (proliferation marker) in these cells [27]. The most important observation made in the present study was the ability of *YK* to synergize with the action of paclitaxel - a widely used anticancer drug. Since most anticancer therapies act by induction of apoptosis which often lead to resistance, the combinatorial treatment could be advantageous as a potent strategy to bypass resistance [28]. The synergy between *YK* and paclitaxel was seen at all levels including the inhibition of cell cycle progression and even activation of p53 (Figure 2C). Angiogenesis is a key requirement for tumorigenesis and blocking the process appears to be an effective strategy to combat cancer [29]. Many tumors show increased expression of VEGF compared to normal tissues [30]. Therefore, therapies directed against VEGF or its receptors hold great promise in cancer treatment. Incidentally, *YK* treatment also led to a reduction in VEGF secretion by cancer cells indicating the anti-proliferative signaling by *YK* (Table 1). Since the analytical profiling of *YK* reproducibly showed the presence of some specific components in this formulation (Additional file 1: Figure S1), it will be desirable to study each molecular component of this formulation to understand the pharmacological principles of *YK*.

## Conclusions

*YK* is an ovarian cancer-specific and effective traditional Tibetan formulation bearing the following anticancer properties: (i) imposes G1 arrest of cells by activating p53, (ii) induces cytochrome c release from mitochondria, and (iii) inhibits angiogenesis. Further, *YK* could be of immense pharmacological significance as it complements the action of known anticancer drugs like paclitaxel which may allow improving the efficacy and potency of conventional drugs and reduce side effects. Thus, *YK* appears to be a strong candidate as novel therapeutic for the ovarian cancer patients.

## Electronic supplementary material

Additional file 1: Figure S1: Analytical profile of *Yukyung Karne (YK)*. YK sample (300 mg in water) was analyzed by reverse phase-HPLC (Shimadzu) on a C18 column using 2% acetonitrile gradient from 5% to 95% over a 55 minute run (flow rate of 1.0ml/min). Sample detection was done at 220 and 280nm under ambient temperature conditions. (PDF 48 KB)

## Abbreviations

DMEM: Dulbecco-modified Eagle’s medium
ECL: Enhanced chemiluminescence
FBS: Fetal bovine serum
MTT: 3-[4,5-dimethylthiazol-2-yl]-2,5 diphenyltetrazolium bromide
TTM: Traditional Tibetan medicine
TUNEL: Terminal deoxynuleotidyl transferase dUTP nick end labeling
VEGF: Vascular endothelial growth factor
YK: Yukyung Karne.
